This article has been retracted.

# Green Finance Evaluation Based on Neural Network Model

**DOI:** 10.1155/2022/4803072

**Published:** 2022-08-17

**Authors:** Ke Wang

**Affiliations:** School of Economics and Management, Huzhou College, Huzhou, Zhejiang 313000, China

## Abstract

The weights of green finance indicators are established in accordance with the AHP in order to suggest an evaluation system that is more thorough and reasonable and to construct an evaluation index system. The findings indicate that the growth of urban green finance is more closely correlated with the development of environmental protection businesses, capital allocation efficiency, and governmental and social capital support. Regulation of consumption also has a significant impact. In order to encourage the growth of urban green finance, this paper analyzes the scoring outcomes and changes for each city and offers solutions and recommendations.

## 1. Introduction

In recent years, from the proposal and research of green finance to the implementation of policy recommendations, it has received extensive attention from all parties. Improving the green financial system has become the common understanding of every country at present. The green finance development strategy has become China's national strategy.

Nowadays, the concept of green finance has been widely recognized by all sectors of society; the research results are increasing day by day; and most of them focus on the discussion of connotation concepts, product and tool innovation, policy mechanisms, and practical experience promotion [1]. However, its development is relatively slow; in the final analysis, there are still many problems in the green financial system. Foreign research on green finance is earlier, and the system is relatively mature. The research on the evaluation system involves macro- and microlevels [2, 3]. It started late in China; the development of green finance is not high; and the popularity is not enough. In addition, due to the differences in domestic and foreign economic environments, the practical experience of foreign green finance has limited reference to the development of China's green finance. Therefore, it is necessary to construct a standard evaluation system with universal applicability to quantify the development level and stage of green finance [4, 5]. Green finance is a financial innovation based on the concept of sustainable economic and social development in the financial industry. Its advanced nature is reflected in the combination of economic and social benefits, and the incorporation of environmental factors into the evaluation system of economic development [6]. After years of economic development in China at the expense of the environment, environmental problems have begun to plague people's lives, and green development is particularly important. In addition, the gradual slowing economic growth trend under the new normal indicates that China can no longer rely on its resource advantages for extensive development, and the transformation of the economic structure and the optimization and upgrading of the industrial structure are imminent.

Since the concept of green finance was put forward, many economic scholars have conducted in-depth research on the evaluation and application of green finance. For example, Wang et al. [7] predicted the green finance index and development according to the characteristics of China's green finance. Sun [8] used the neural network to study the correlation between green finance and carbon emissions. Li and Gan [9] and Huang and Chen [10] studied the correlation between ecological environment development and green finance, and proposed the ecological issues to be solved by green finance; He et al. [11] studied the relationship between green finance and smart city development, and proposed to lead the urban ecological construction through green finance. Green finance is a new model proposed for the establishment of environmental protection. It belongs to a major innovation in the financial system [12]. Green finance affects the current domestic production of green factors, which is in line with the current direction of national environmental protection and sustainable development [13]; the green finance policy integrates the current internet technology and applies a variety of technical means to achieve the sustainable development of green finance [14]. Lv et al. [15] studied the development strategies of green finance with different regional characteristics in China. Due to the different regional economies, there are differences in the green finance strategies formulated by government departments. Jiang et al. [16] proposed a green finance index system based on an improved entropy model and applied these index systems to forecasting in some common economic fields. Green finance is closely related to the current development direction of China's low-carbon economy, and its concepts and policies are helpful to promote the development of China's current low-carbon economy [17, 18].

G20 leaders proposed seven optional measures at the 2016 Hangzhou summit, emphasizing the need to “develop green finance.” Growing in importance is the role that green finance plays in advancing China's economic growth. Policies have guaranteed the development of green finance and supported it with resources such as talent, materials, and technology [19]. According to the G20 summit's questionnaire to the IFC, the majority of green finance indicators are only created for specific financial products or markets, and there is a lack of a more comprehensive and more scientific green finance measurement and evaluation indicator system. A new type of green finance index evaluation tool is established by using the neural network model in response to the current situation, which is that the green finance evaluation system, both domestically and internationally, is not yet perfect. A few regions in the northwest are severely polluted by industrial emissions, so their goal should be to take action to reduce pollution. Some regions along the southeast coast, for instance, have high energy consumption, so the focus of future development should be on reducing energy consumption. In this way, the role of reducing resource waste rate, etc., in the countermeasures against climate change, can make the services of green finance achieve high quality on the basis of perfection. We encourage the use of financial instruments and policies that are related to supporting the transition of the economy to a green one, improving the environment in which green finance can operate, setting up a reliable information system for evaluation, stepping up oversight of the sector, and reducing and resolving risks associated with it. In order to significantly speed up the development of green finance, research on the subject is being performed using a neural network model to evaluate green finance.

## 2. The Concept of Green Finance

The three categories of green finance principles that the current theoretical framework allows for are explained below. First, looking at it through the lens of economic theory, by increasing the cost of pollution and decreasing the cost of environmental protection projects, making money available for investment in green industry economies and projects can influence people to choose green consumption and behavior [20]. Second, from the viewpoint of ecological economics, the risks associated with the use of environmental resources by economic entities are converted into value through the market, such as the market for carbon trading. Finally, from a methodical standpoint, we consider financial activities and the environment as a whole while revealing and evaluating the interaction between finance and the environment using green information systems. From this vantage point, green finance is related to but distinct from traditional finance. In order to encourage green development, finance engages in a set of behaviors that reflect green concepts in financial activities. Thus, the definition of “green finance” in this paper refers to a financial business model that takes this relationship into account.

Financial institutions and businesses are typically the main actors in green finance projects. Financial institutions' nature still compels them to pursue profits as their ultimate objective. As a result, there have been long-running discussions in theoretical circles about how to balance and select between the two. In reality, the objective is to maximize profits because failing to do so increases the risk of it becoming difficult to survive. Therefore, by implementing policies from top to bottom, the government and pertinent regulatory bodies need to address the market failure brought on by externalities.

## 3. Green Finance Evaluation Index System

The discussion of green finance at the moment, both domestically and internationally, is primarily at the qualitative level, which is comparatively more theoretical, such as connotation definition, policy system, and mechanism of action. The nature of green finance involves a wide range, and the definition is relatively complex, so there is not enough quantitative research in evaluation research due to the high difficulty of data collection, the lack of related studies on quantitative evaluation and quantitative research on specific indicators, and the fact that the market is not perfect in terms of systems, programs, etc.

### 3.1. Indicator Selection Principle

#### 3.1.1. Scientific and Rational

Green finance must be developed, economic development and ecological protection must have both, and ecological construction is the development of green finance.

The basic requirement is that economic development is the core purpose of green finance. Only by taking these two points into consideration can a conformity be established in the scientific system. The premise of ensuring that the evaluation results are objective and reasonable is the selection of indicators.

In the process, the indicators are selected in a scientific and reasonable way, and at the same time, they hold a scientific attitude and grasp the law of development. When dividing dimensions, paddling should be realistic. When selecting relevant indicators, the data sources should be authentic and reliable, and Qinghai should also be considered.

The construction is more scientific and reasonable.

#### 3.1.2. Feasibility and Measurability

When establishing an indicator system, it must be rooted in the theoretical soil of green finance, and indicators must be refined and refined.

It cannot be ambiguous to avoid misunderstandings when screening, collecting, and interpreting indicators. At the same time, it must be measurable, which it requires that the selection of green finance development indicators can go deep into the connotation of green finance, and cannot only see its appearance's present form. Second, the evaluation indicators should preferably be realistic and can be used in the practice of green financial activities.

To ensure that data can be obtained directly from authoritative sources such as national or local, or, through existing authoritative statistics, the data are converted to ensure the feasibility and measurability of the index measurement.

#### 3.1.3. Representation and Authority

The design of the green finance indicator system aims to more accurately reflect the state of green finance development in Qinghai. However, there are a lot of overlapping, related, or overlapping elements among them. All indicators can be included in the evaluation system if completeness is the only factor taken into account, but this will make the evaluation system bloated, ineffective, and low. Therefore, the chosen index should be both representative and authoritative in order to avoid the issue of low efficiency while guaranteeing the quality of index evaluation. Additionally, we must stop using the indicators that are still up for debate and work to represent the most comprehensive evaluation system with the fewest possible indicators. Finally, representative indicators should more accurately reflect the historical state of green finance development while also serving as a foundation for future directions in improvement.

#### 3.1.4. Systematic and Comprehensive

The growth of regional green finance has a wealth of content and has the potential to become an independent system. The development of green finance in our nation is currently dependent more on raising the caliber of green financial services than it is on spreading the idea of financial green. To effectively reflect the effects of green finance across various industries and time periods, the indicator system's design should take the level of green financial services into account. Green credit holds a significant position within the field of green financial services at this point, which includes many areas such as credit, insurance, and securities. The indicator design thus demonstrates the continued requirement to reflect the preeminent role of banking financial institutions in green finance. In addition, by combining various dimensions and indicators, such as securities, insurance, investment, and trading, we can view a systemic problem like the development of green finance from a thorough and comprehensive angle.

#### 3.1.5. Comparability and Independence

In this study, green finance is a macro concept, and its evaluation system does not exist in isolation. It is impossible to draw accurate conclusions by measuring the development of green finance alone without making comparisons. To form an indicator system, it is necessary to pay attention not only to the continuity in time, but also to the differences in regions, and to avoid the strong correlation between various elements, so as to measure the development level of green finance more accurately.

### 3.2. Selection of Green Finance Evaluation Indicators

The selection of indicators starts from a macro perspective and takes into account the above two. Therefore, according to the relevant literature, the relevant indicators were screened and summarized as shown in Table 1.

### 3.3. Indicator Data Source

The indicator data involved come from wind, business databases, or public yearbooks. For the data that cannot be directly obtained, most of them are obtained by adding subdivided indicators, or using formulas to calculate, or using alternative indicators to represent their data. For situations where green credit data did not exist before 2012, we consider using credit as an alternative to investment quotas for green industries and green projects. If there are no relevant data that cannot be replaced, it is measured with a value of 0 for data analysis. The data of each indicator are provincial-level data. If there is no relevant statistical value, it can be obtained by calculating other indicators.

### 3.4. Determination of the Weight of Green Finance Evaluation Indicators

#### 3.4.1. Data Standardization Processing

It is necessary to standardize the original data in order to eliminate differences between features and make all features have the same scale due to variations in the measurement units used by the different indicators in the indicator system. Therefore, different normalization treatments are used for positive and negative indicators.

Positive indicators are as follows:

(1) $$\begin{array}{c} Z_{ij}=\frac{X_{ij}-\text{min}\left\{X_{1j},\ldots ,\right\}}{\text{max}\left\{X_{1j},\ldots ,X_{nj}\right\}-\text{min}\left\{X_{1j},\ldots ,X_{nj}\right\}}. \end{array}$$

Negative indicators are as follows:

(2) $$\begin{array}{c} Z_{ij}=\frac{\text{max}\left\{X_{1j},\ldots ,X_{nj}\right\}-X_{ij}}{\text{max}\left\{X_{1j},\text{…},X_{nj}\right\}-\text{min}\left\{X_{1j},\ldots ,X_{nj}\right\}}, \end{array}$$

where *X*_*ij*_ represents the value of the *j*-th index of the *i*-th sample in the evaluation system of *n* samples and *m* indicators (*i* = 1, 2,…, *n*; *j* = 1, 2,…, *m*), and *Z*_*ij*_ represents normalized data.

#### 3.4.2. Entropy Weight Method to Determine Index Weight

The principle is to measure its comparative effect on the system according to the discrete degree of the index data, that is, the amount of effective information, so as to give the index a certain weight. The greater effectiveness of the information contained, the greater its impact on it, so the weight is given. Specific steps are as follows:

The ratio of the *i*-th sample value under the *j*-th indicator to the indicator is as follows:

(3) $$\begin{array}{c} P_{ij}=\frac{X_{ij}}{\sum_{i=1}^{n}X_{ij}}，\\ i=1,2,\ldots ,n,\\ j=1,2,\ldots ,m. \end{array}$$

(a) We calculate the entropy value of the *j*th indicator as follows:
  (4) $$\begin{array}{c} e_{i}=-k\sum_{i=1}^{n}P_{ij}\text{ln}\left(p_{ij}\right),\\ j=1,2,\ldots ,m, \end{array}$$
Among them, *k*=(1/ln(*n*)) > 0,  satisfying *e* ≥ 0
(b) We calculate the redundancy (difference) of information entropy as follows:
  (5) $$\begin{array}{c} d_{i}=1-e_{j},\\ j=1,2,\ldots ,m. \end{array}$$
(c) We calculate the weight of each indicator as follows:
  (6) $$\begin{array}{c} w_{j}=\frac{d_{j}}{\sum_{j=1}^{m}d_{j}},\\ j=1,2,\ldots ,m. \end{array}$$

The weight setting value involved in the evaluation can be obtained from the previous calculation formula, which is the result shown in Table 2.

The total amount of foreign capital utilization, the share of businesses engaged in environmental protection in total enterprise value, and the efficiency of loan allocation all account for significant weight in the weight results measured using the entropy weight method, as shown in Table 2. These values, which are 0.1333, 0.1043, and 0.0877, respectively, show that the level of development of urban green finance has a significant impact. The proportion of solid waste emission per unit of GDP, the market value of energy-consuming enterprises, and energy consumption per unit of GDP are small and have a significant impact on the development of urban green finance, which are 0.0326, 0.0387, and 0.0390, respectively.

## 4. Green Finance Evaluation Based on Neural Network Model

### 4.1. Neural Network Model

A popular machine learning model [21] called a neural network [22] has been extensively used in a variety of economic and industrial sectors to complete business prediction and evaluation through data mining and analysis. By transmitting signals between the topological structures of the neural network forward and the error between the topological structures backward, the model continuously modifies the weights and thresholds of the network, reducing the error of a single sample and ultimately causing the total error *E* to tend toward the minimum. Its formula is as follows:

(7) $$\begin{array}{c} E_{k}=\frac{1}{2}\sum_{j=1}^{M}{\left(d_{j}-Y_{j}\right)}^{2},\\ E=\sum_{k=1}^{K}E_{k}=\frac{1}{2}\sum_{k=1}^{K}\sum_{j=1}^{M}{\left(T_{j}^{k}-Y_{j}^{k}\right)}^{2}, \end{array}$$

Among them, *E*_k_ is the training sample error, *M* is the number of units in the set output layer, *d*_j_ is the target value of the unit *j* to the training sample, *Y*_j_ is the output value of the training sample, and *E* is the total error calculated by the neural network.

Training and testing are both a part of the BP neural network's prediction of urban green finance. The process is as follows: first, we gather knowledge from training samples, then store network weights and threshold information, then input testing samples, and finally, compare predicted and actual output. A comparison check is performed on the result. In this paper, a three-layer structure is chosen. The input layer contains 15 nodes, which is consistent with the number of indicators of the level of urban green development. The output layer contains 1 node, which represents the score of urban green financial development. There is no widely accepted, simple theory for identifying the layers. The empirical formula for the hidden layers chosen for this study is as follows:

(8) $$\begin{array}{c} H=\frac{a+b}{2}, \end{array}$$

where a is the number of input layers and *b* is the number of output layers. It can be known from equation (8) that the number of hidden layers selected in this paper is 8, so the topology of the neural network model is 15-8-1.

### 4.2. BP Neural Network Process

Figure 1 depicts how the BP neural network model was used to evaluate green finance. In order to obtain standardized data, the evaluation index values for a particular location are first collected or input. The neural network model initializes the length of the BP neural network weight threshold to obtain the ideal weight threshold, calculate the evaluation error in accordance with the model rules, and then update the neural network structure in accordance with the evaluation requirements. The weight threshold is used to determine whether the end condition has been satisfied after these values have been updated. The final evaluation result is shown upon fulfillment of the end condition. Otherwise, the cycle moves on to the stage where the weight threshold update is determined and the optimal weight threshold is once again acquired.

## 5. Experimental Analysis

### 5.1. Predictive Analysis of BP Neural Network

A province's urban green finance development level was measured using 42 groups of indicator data in 2019 and 2020; 36 groups were chosen as training samples, and 6 groups served as samples for the prediction test. There are 21 cities, numbered C1, C2,…, C21, and the index data for each are set as the input data for the BP neural network. Each city's score can be determined using. The population size is 20, the number of evolutionary generations at their most is 20, the probability of crossover is 0.8, and the likelihood of mutation is 0.1, using a neural network interface for training. The test results are depicted in Figure 2, where the average error percentage is 0.4035 percent and the maximum error percentage is 1.4236 percent.

The outcomes demonstrate that the neural network model's prediction error is lower and that its prediction of the level of urban green finance development is more accurate. As a result, the BP neural network evaluation model is chosen for the evaluation of green finance.

### 5.2. Green Finance Single Indicator Analysis

Energy consumption per unit of GDP (10,000 tonnes of standard coal/100 million yuan) and “market value ratio of high energy-consuming enterprises” were chosen as the two indicators to test the effect of a single indicator on the evaluation score of green finance. C1, C2, C7, and C19 were the selected cities for comparison. Energy consumption as a percentage of GDP is measured in units of “10,000 tonnes of standard coal/100 million yuan” and “the proportion of the market value of high energy-consuming enterprises” as a percentage. Figures 3 and 4 compare various measures of energy consumption per unit of GDP and the market value of businesses with high energy consumption, respectively.

Figures 3 and 4 show that the proportion of the tertiary industry in C1 and C2 cities is relatively high, which is intuitively obvious. It is possible to hasten economic development by developing the tertiary sector. The output value and the number of units in the two cities' high-energy industries are also relatively low, suggesting that these cities control the growth of businesses with “two highs and one surplus.” Social funds are thus distributed to specific environmental protection fields and projects. However, C2's unit GDP power consumption and energy consumption scores are both low, demonstrating the C2 economy's heavy reliance on energy and the need to improve the structure of energy consumption. It helps green businesses increase their access to financing; however, green credit still needs to be improved in order to raise the overall bar for green finance. Green finance development levels in C7 and C19 need to be raised, and the green securities' indicators of C1 are advantageous in showing that the security industry is healthy and environmentally friendly. Although the level of financial development is low compared to the proportion of the C7 tertiary industry, more money should go toward this sector. The industrial waste gas and waste emissions of C19 remain extremely high when viewed from the perspective of the proportion. Businesses that do not abide by national industrial and environmental protection policies will be encouraged to change their industrial structures by the implementation of industrial and environmental protection policies. It will also advance the advancement of green insurance by raising awareness of environmental liability insurance throughout the entire society.

## 6. Conclusions and Countermeasures

### 6.1. Adhere to Two-Pillar Regulation

“Dual pillar” refers to strengthening the emphasis on macro-prudential policy and monetary policy, while the financial development system is oriented toward high-level and high-quality development, which determines that green finance, an important strategic part of finance, should improve its quality, that is, green financial institutions not only epitaxial growth, but also high-quality endogenous growth.

### 6.2. Innovate Green Financial Products and Services

We resolutely prevent the occurrence of systemic financial risks; promote the innovation of a green credit system closely integrated with environmental protection; make full use of the concept of green environmental protection in the process of policy introduction, business promotion, and product design; establish environmental protection and low consumption funds; actively promote low-carbon economic projects; and establish a market-oriented green technology innovation system.

We increase capital's support for enterprises. The government guides social capital to flow into green industries and plays a role in financial innovation. Through innovative financial tools such as green credit, it expands financing channels for green industries in multiple ways and from multiple perspectives, and supports the growth of small and microenterprises. We promote environmental protection and energy-saving innovation, develop a circular economy, and realize the upgrading of urban industrial structure.

### 6.3. Provide a Favorable Market Environment for Promoting Green Finance Evaluation

We create a system to enhance the green financial market and green financial evaluation from the virtual to the real. The real economy should benefit from and be inseparable from the green financial evaluation. To foster a positive interaction with the real economy, the two should be concurrently developed and be in complete coordination. The green financial market supervision and service departments should strengthen their roles, fully absorb advanced knowledge from abroad, and inject vitality into the system's improvement. This shift from emphasizing speed of development to improving the quality of development is necessary.

We enhance the effectiveness of financial capital allocation, reinforce the government's active oversight role in the flow of financial resources to green industries, lower the entry barrier to the market, boost market vitality, and enhance the market's capacity for resource allocation. We enhance the mechanism for removing outdated production capacity; strengthen the direction of industrial policies; fully utilize the functions of the departments of investment management, environmental protection, quality control, and other enterprises; encourage and support the growth of advanced production capacity; and promote the orderly industrial ecological transformation.

### 6.4. Increase the Disclosure of Information in Green Finance Evaluation

We promote the orderly development of green finance evaluation platforms, increase disclosure, and expand the channels for sharing information by expanding the channels of information communication for green finance in the evaluation process and results. We improve the data on green finance and the openness with which information is disclosed, laying the groundwork for the creation of a system for evaluating green finance that is more thorough. We create a green financial platform, broaden the distribution of green financial information, create green financial information services, lower the cost of information for investors, and encourage more investors to invest in regional green projects. We create a mechanism for green finance cooperation, make investments in regions with better resource agglomeration effects, play up the green finance diffusion effect, and encourage the spread of financial capital to nearby regions with low-value resources to advance the development of finance as a whole.

## Figures and Tables

**Figure 1:** Green finance evaluation process based on the BP neural network model.

**Figure 2:** Prediction of green finance evaluation scores under the BP neural network.

**Figure 3:** Comparative analysis of indicators of energy consumption per unit of GDP.

**Figure 4:** Comparative analysis of the market value of high energy-consuming enterprises.

**Table 1:** Green finance indicator system.

Criterion layer	Indicator layer	Indicator meaning
Environment	Industrial wastewater discharge/city GDP	Wastewater discharge per unit of GDP (10,000 tonnes/100 million yuan)
	Exhaust emissions per unit of GDP (10,000 cubic meters/100 million yuan)	Industrial exhaust emissions/city GDP
	Solid waste discharge per unit of GDP (10,000 tonnes/100 million yuan)	Industrial solid waste production/urban GDP
	Energy consumption per unit of GDP (10,000 tonnes of standard coal/100 million yuan)	Total industrial energy consumption/urban GDP

Finance	Deposit ratio	Total loans of financial institutions at the end of the year/total deposits of financial institutions at the end of the year
	Savings rate	Year-end total deposits of financial institutions/GDP
	Market value of environmental protection companies	Gross output value of environmental protection enterprises/A-share market value
	Proportion of market value of high energy-consuming enterprises	The total market value of the six high-energy-consuming enterprises/A-share market value

Society	Insurance depth	Premium income/GDP
	Loan allocation efficiency	The proportion of urban GDP in the province/the proportion of local loans in the province
	Total foreign investment and utilization (100 million yuan)	The actual utilization of foreign investment
	Marginal capital productivity	Gross economic growth/gross capital formation
	Proportion of environmental protection investment	Environmental protection investment/GDP
	Proportion of public expenditure on energy conservation and environmental protection	Financial expenditure on energy conservation and environmental protection/total financial expenditure
	Proportion of transaction volume of CDM projects	Number of clean energy projects/number of local projects

**Table 2:** Analysis results of the entropy weight method.

Index	Weights	Index	Weights
Wastewater discharge per unit of GDP	0.0525	Proportion of environmental protection investment	0.0768
Exhaust emissions per unit of GDP	0.0474	Proportion of public expenditure on energy conservation and environmental protection	0.0514
Solid waste per unit of GDP	0.0326	Clean development mechanism project	0.0614
Waste emissions	0.0390	Transaction volume ratio	0.1333
Energy consumption per unit of GDP	0.0877	Total utilization of foreign investment	0.0688
Loan allocation efficiency	0.066 1	Deposit ratio	0.0703
Insurance depth	0.0387	Savings rate	0.0697
Proportion of market value of high energy-consuming enterprises	0.1043	Marginal capital productivity	0.0514
Market value of environmental protection companies	0.0474		

## Data Availability

The data used to support the findings of this study are available from the corresponding author upon request.

## References

[1] Taghizadeh-Hesary F., Yoshino N. (2019). The way to induce private participation in green finance and investment. *Finance Research Letters*.

[2] Ng A. W. (2018). From sustainability accounting to a green financing system: institutional legitimacy and market heterogeneity in a global financial centre. *Journal of Cleaner Production*.

[3] Zhang D., Mohsin M., Rasheed A. K., Chang Y., Taghizadeh-Hesary F. (2021). Public spending and green economic growth in BRI region: mediating role of green finance. *Energy Policy*.

[4] Zheng Y., Ye X. (2022). An evaluation model of an urban green finance development level based on the GA-optimized neural network. *Mathematical Problems in Engineering*.

[5] Wang X., Wang Q. (2021). Research on the impact of green finance on the upgrading of China’s regional industrial structure from the perspective of sustainable development. *Resources Policy*.

[6] Wen G., Xiaohang M., Yingjie Q., Yuiu W. (2019). Financial supply-side structural reform in China: with special reference to green finance. *International Information Institute (Tokyo)*.

[7] Wang X., Zhao H., Bi K. (2021). The measurement of green finance index and the development forecast of green finance in China. *Environmental and Ecological Statistics*.

[8] Sun C. (2021). The correlation between green finance and carbon emissions based on improved neural network. *Neural Computing & Applications*.

[9] Li C., Gan Y. (2021). The spatial spillover effects of green finance on ecological environment—empirical research based on spatial econometric model. *Environmental Science and Pollution Research*.

[10] Huang Y., Chen C. (2022). The spatial spillover and threshold effect of green finance on environmental quality: evidence from China. *Environmental Science and Pollution Research*.

[11] He Z., Liu Z., Wu H., Gu X., Zhao Y., Yue X. (2020). Research on the impact of green finance and Fintech in smart city. *Complexity*.

[12] Huang H., Zhang J. (2021). Research on the environmental effect of green finance policy based on the analysis of pilot zones for green finance reform and innovations. *Sustainability*.

[13] Lee C.-C. (2022). How does green finance affect green total factor productivity? Evidence from China. *Energy Economics*.

[14] Wang K., Tsai S. B., Du X., Bi D. (2019). Internet finance, green finance, and sustainability. *Sustainability*.

[15] Lv C., Bian B., Lee C. C., He Z. (2021). Regional gap and the trend of green finance development in China. *Energy Economics*.

[16] Jiang L., Wang H., Tong A. (2020). The measurement of green finance development index and its poverty reduction effect: dynamic panel analysis based on improved Entropy method. *Discrete Dynamics in Nature and Society*.

[17] Zhang W., Zhu Z., Liu X., Cheng J. (2022). Can green finance improve carbon emission efficiency?. *Environmental Science and Pollution Research International*.

[18] Li W., Fan J., Zhao J. (2022). Has green finance facilitated China’s low-carbon economic transition?. *Environmental Science and Pollution Research International*.

[19] Berensmann K., Volz U., Alloisio I. (2017). Fostering sustainable global growth through green finance–what role for the G20. *T20 Task Force on Climate Policy and Finance*.

[20] Dikau S., Volz U. (2021). Central bank mandates, sustainability objectives and the promotion of green finance. *Ecological Economics*.

[21] Cai W., Gao M., Jiang Y. (2022). Hierarchical domain adaptation projective dictionary pair learning model for EEG classification in IoMT systems. *IEEE Transactions on Computational Social Systems*.

[22] Li J., Chen Z., Cheng L., Liu X. (2022). Energy data generation with wasserstein deep convolutional generative adversarial networks. *Energy*.

